# Design of an Intelligent Nursing Information Management System for Critically Ill Patients in Neurosurgery

This article has been retracted.

**DOI:** 10.1155/2022/2848255

**Published:** 2022-04-04

**Authors:** Hongrong Wang, Yan Liu, Fang Liu

**Affiliations:** ^1^Emergency Department, The Affiliated Yantai Yuhuangding Hospital of Qingdao University, Yantai, China; ^2^Department of Nursing, Dongying People's Hospital, Dongying, China; ^3^Neurosurgery Department, The Affiliated Yantai Yuhuangding Hospital of Qingdao University, Yantai, China

## Abstract

In hospitals, one of the dominant issues is the development of an accurate and precise nursing management system which is hard to implement due to the various problems in the implementation of the traditional manual system. For this purpose, we are to solve the imperfect functions of the traditional nursing information management system and the strong subjectivity and low accuracy of the way of manually judging the patient's condition. Firstly, the Immune Genetic Algorithm (IGA) is used to optimize the Backpropagation Neural Network (BPNN). A mortality prediction model using IGA-BPNN is proposed. Secondly, a nursing information management system for critically ill patients in neurosurgery is designed. The IGA-BPNN prediction model is used as a part of the system to predict the mortality of critically ill patients. Finally, the performance of the predictive model and the system is tested using the Medical Information Mart for Intensive Care (MIMIC)-III data set design experiment. The results show the following: (1) Precision, Recall, and *F*1-score of mortality prediction using the IGA-BPNN model are 7.2%, 7.2%, and 7.3% higher than those of other prediction models. The designed model has better performance. (2) The comprehensive performance of the system during operation can reach the standard. The researched content aims to provide important technical support for the nursing information management of critically ill patients in neurosurgery and the intelligent analysis of patients' condition.

## 1. Introduction

The main types of patients admitted to the Neurological Intensive Care Unit (NICU) are critically ill patients of the nervous system. The ward is mainly used for the recovery of patients after neurosurgery, the treatment of critically ill patients, and the rescue of emergency patients, and so on [1]. Therefore, when the special functions of the NICU are used, it must focus on efficiency. In this process, it is very important to seek standardized, rationalized, and scientific management methods [2]. At present, the hospital's NICU still has serious problems such as uneven construction level, irregular patient admission, and management confusion, which will undoubtedly lead to delays in patients' conditions and even medical accidents [3]. Doctors diagnose and treat patients using their basic information, cases, and monitoring information. If effective methods are not used to manage the patient's care information, it will greatly increase the disability and mortality of patients.

The Internet has become an indispensable tool in people's lives and work. The promotion of the information management system in the hospital has greatly reduced the cost of manpower and material resources and strengthened the collaboration of various positions, ranks, and departments [4]. Cao and Zhu carried out a modular design for the pediatric nursing information management system. Visual FoxPro 5.0 was used for programming, and the clinical pediatric care information system was tested. The results have shown that the system optimizes the pediatric nursing process, improves the work efficiency of medical staff, and greatly reduces the loss of medical records, errors, and supervision problems [5]. Shahmoradi et al. investigated the use of the Hospital Information System (HIS) standard in the Tehran University of Medical Sciences Hospital and found that the HIS system structure is not standardized [6]. Explanation: although HIS can bring great convenience to medical staff, there are still irregularities in its construction and use. Nursing information system is an important part of HIS. It only provides the functions of query, entry, and deletion of basic patient information and diagnosis and treatment data and cannot analyze this information to assist doctors in diagnosis and treatment [7]. Therefore, it is necessary to adopt some analytical techniques to improve the nursing information management system.

Under normal circumstances, doctors are using their own experience and then using the patient's relevant diagnosis and treatment information to judge their condition. This has high requirements on the doctor's own ability and has the defects of strong subjectivity and low accuracy. Firstly, the Immune Genetic Algorithm (IGA) is used, and the Backpropagation Neural Network (BPNN) is optimized. A mortality prediction model using IGA-BPNN is proposed. Secondly, a nursing information management system for critically ill patients in neurosurgery is designed. The IGA-BPNN prediction model is used as a part of the system to predict the mortality of critically ill patients. It assists the doctor to accurately judge the patient's condition through intelligent means. Finally, the performance of the experiment on the prediction model and the system is tested.

One of the dominant issues is the development of an accurate and precise nursing management system, which is hard to implement due to the various problem in the implementation of the traditional manual system. For this purpose, we are to solve the imperfect functions of the traditional nursing information management system and the strong subjectivity and low accuracy of the way of manually judging the patient's condition. Firstly, the Immune Genetic Algorithm (IGA) is used to optimize the Backpropagation Neural Network (BPNN). A mortality prediction model using IGA-BPNN is proposed. Secondly, a nursing information management system for critically ill patients in neurosurgery is designed. The IGA-BPNN prediction model is used as a part of the system to predict the mortality of critically ill patients. Finally, the performance of the predictive model and the system is tested using the Medical Information Mart for Intensive Care (MIMIC)-III data set design experiment. The purpose of the research is to provide important technical support for the nursing information management of critically ill patients in neurosurgery and the intelligent analysis of the patient's condition.

The rest of the paper is organized as given below.

In the section entitled “Proposed Methodology,” Immune Genetic Algorithm along with optimization algorithm, that is, Backpropagation Neural Network, is described in detail. Moreover, these algorithms are combined to form a hybrid and more accurate prediction model to resolve the issue under consideration in this paper. Experimental results and observations were presented to verify effectiveness of the proposed hybrid model in realistic environment of hospitals. A discussion section is provided to discuss how the scheme is developed and how it is effective in solving the issue. Finally, summarized form of the proposed scheme along with the referencing materials is provided in the last section of the manuscript.

## 2. Proposed Methodology

### 2.1. System Key Technology Analysis

#### 2.1.1. System Architecture

Currently, Client-Server (C/S) and Browser-Server (B/S) system architectures are widely used. In the C/S architecture, firstly, the request sent by the user to the system is submitted by the Client program to the Server program. The Server program handles the request accordingly and returns the processing result to the Client program. Finally, the Client program is used to present the results in a certain form to the user. The C/S architecture has strong transaction processing capabilities and data manipulation capabilities, and its structure is simple and easy to operate. However, the development cost, software maintenance cost, and upgrade difficulty of the C/S architecture also increase as the complexity of the system software gradually increases [8].

The B/S architecture is an improvement of the C/S architecture, in which system users mainly perform corresponding operations in the browser. The main transaction is performed on the server, and the rest of the small part of the transaction is performed on the browser. This mode undoubtedly greatly reduces the burden on the client computer and reduces system maintenance and upgrade costs to a certain extent. However, the B/S architecture is far inferior to the C/S architecture in terms of the response speed of data query and statistics, and its software expansion capability is poor, and its security is also low [9]. The advantages and disadvantages of the two system architectures are compared in Table 1 [10].

In Table 1, the B/S architecture and the C/S architecture have their own advantages and disadvantages. Therefore, the adoption of the B/S-C/S hybrid system architecture will give play to its greatest advantages in the design of the nursing information management system.

#### 2.1.2. Network Architecture

The network of this system is mainly composed of central monitoring station, intensive care workstation, wireless router, and mobile terminal, as shown in Figure 1.

Each bed in the neonatal intensive care unit (NICU) ward is equipped with 4 network ports. The central acquisition mode is adopted, the equipment is connected to the switch through the local area network, and the patient's information is centrally collected through a central monitoring system host. Each hospital bed is equipped with a computer as an intensive care workstation. The wireless router is placed on the top of the NICU ward to achieve full coverage of the wireless network of the entire ward. Mobile devices placed next to the hospital bed can connect to the server through the wireless network.

#### 2.1.3. Oracle Database

Oracle database is the most widely used database management system in the world. It mainly consists of three types of files: database files, log files, and control files. As a general database system, it has complete management functions and distributed processing functions. Oracle database has four main features in function: (1) It can support a large number of users to perform various operations on the same database and can ensure data consistency through the database lock mechanism. (2) It can provide access criteria for ensuring the security of the database, data changes are synchronized, and the data logic and physical independence are independent criteria. (3) The distributed processing function of the oracle database can largely ensure data consistency and location transparency. (4) The database can process and manage a large amount of data in a unified manner to achieve the purpose of efficiently accessing a large amount of data [11].

The nursing information management system needs to deal with many data information, reports, and data statistics exporting about the patient's condition every day. Therefore, a secure, stable database with huge data processing functions plays an important role in the system. Oracle database can handle these problems very well. Therefore, it is used as the database behind the nursing information management system.

### 2.2. Mortality Prediction Model Using IGA-BPNN

#### 2.2.1. Improved BP Algorithm

BP neural network is a multilayer feedforward network trained according to the error backpropagation algorithm. It is one of the most widely used neural network models [12]. The BP network can learn and store a large number of input-output mode mapping relationships. There is no need to reveal the mathematical equation describing this mapping relationship in advance [13]. BPNN is a multilayer perceptron structure, which mainly contains an input layer, a hidden layer, and an output layer [14]. The BPNN structure is shown in Figure 2.

In Figure 2, BP neural network only contains one input layer, one output layer, and several hidden layers. The external information is imported into the model through the input layer, processed layer by layer in the hidden layer, and finally output the result in the output layer [15]. The input layer and the output layer are directly connected with the outside world. Although the hidden layer needs to communicate with the outside world through the above two, every change it produces will have a certain impact on the input layer and output layer. Therefore, the three components of the BP neural network are complementary and inseparable [16]. BP neural network algorithm is abbreviated as BP algorithm, and the specific process is shown in Figure 3.

BP algorithm can transform signal input and output problems into nonlinear optimization problems. Combined with the gradient descent method, an iterative algorithm is used to solve the weights, and the added hidden layer nodes are used to increase the adjustable parameters of the optimization problem, and the optimal solution is expected to be obtained [17]. BP algorithm includes two processes of signal forward and backward propagation in the learning process.

*(1) Forward Transmission*. The forward propagation is carried out from the input layer to the hidden layer and then to the output layer. The input *α*_*i*_ of the *i*th node in the hidden layer can be expressed as

(1) $$\begin{array}{c} \alpha_{i}=\sum_{j=1}^{m}w_{ij}x_{j}+\theta_{i},\;j=1,\;2,\;3,\;\cdots ,\;m, \end{array}$$

where *x*_*j*_ is the input of the *j*th node of the input layer; *w*_*ij*_ is the weight between the *i*th node in the hidden layer and the *j*th node in the input layer; and *θ*_*i*_ is the threshold of the *i*th node in the hidden layer.

The output *β*_*i*_ of the *i*th node in the hidden layer can be expressed as

(2) $$\begin{array}{c} \beta_{i}=\phi \left(\alpha_{i}\right)=\phi \left(\sum_{j=1}^{m}w_{ij}x_{j}+\theta_{i}\right), \end{array}$$

where *ϕ*(*α*_*i*_) represents the activation function of the hidden layer.

The input *δ*_*k*_ of the *k*th node of the output layer can be expressed as

(3) $$\begin{array}{c} \delta_{k}=\sum_{i=1}^{q}w_{ki}\beta_{i}+a_{k}=\sum_{i=1}^{q}w_{ki}\phi \left(\sum_{j=1}^{m}w_{ij}x_{j}+\theta_{i}\right)+a_{k},i=1,\;2,\;3,\;\cdots ,\;q\;, \end{array}$$

where *w*_*ki*_ is the weight between the *k*th node in the output layer and the *i*th node in the input layer and *a*_*k*_ is the threshold of the *k*th node in the output layer.

The output *y*_*k*_ of the *k*th node of the output layer can be expressed as

(4) $$\begin{array}{c} y_{k}=\psi \left(\delta_{k}\right)=\psi \left(\sum_{\mathrm{i=1}}^{q}w_{ki}\beta_{i}+a_{k}\right), \end{array}$$

(5) $$\begin{array}{c} =\psi \left(\sum_{\mathrm{i=1}}^{q}w_{ki}\phi \left(\sum_{\mathrm{j=1}}^{m}w_{ij}x_{j}+\theta_{i}\right)+a_{k}\right), \end{array}$$

where *ψ*(*δ*_*k*_) represents the excitation function of the output layer.

If the error between the actual output signal and the expected output signal is too large, it needs to enter the backpropagation process.

*(2) Backpropagation*. Backpropagation is to pass the output error back layer by layer in the direction of the input layer through the hidden layer and distribute it to all units in each layer and adjust the weight of each unit using the error signal obtained by each layer. Additionally, it will adjust the connection strength and threshold between the input layer, the output layer, and the hidden layer so that the error can be gradually reduced. Continue to repeat this process until the error tends to the allowable range or reaches the preset practice frequency; the learning will be terminated [18]. The quadratic error criterion function *E*_*p*_ for each sample *p* can be expressed as

(6) $$\begin{array}{c} E_{p}=\frac{1}{2}\sum_{\mathrm{k=1}}^{l}{\left(T_{k}-y_{k}\right)}^{2}, \end{array}$$

where *T*_*k*_ represents the expected output and *y*_*k*_ represents the actual output.

The model's total error criterion function for *P* training samples can be expressed as

(7) $$\begin{array}{c} E=\frac{1}{2}\sum_{P=1}^{P}\sum_{\mathrm{k=1}}^{l}{\left(T_{k}^{P}-y_{k}^{P}\right)}^{2}, \end{array}$$

The error gradient descent method is used, and the weights and thresholds of the output layer and the hidden layer are corrected. The weight correction amount Δ*w*_*ki*_ and the threshold correction amount Δ*a*_*k*_ of the output layer is obtained, respectively, as shown in (8) and (9). The weight correction amount Δ*w*_*ij*_ and the threshold correction amount Δ*θ*_*i*_ of the hidden layer are also obtained, as shown in (10) and (11).

(8) $$\begin{array}{c} \Delta w_{ki}=-\eta \frac{\partial E}{\partial w_{ki}}, \end{array}$$

(9) $$\begin{array}{c} \Delta a_{k}=-\eta \frac{\partial E}{\partial a_{k}}, \end{array}$$

(10) $$\begin{array}{c} \Delta w_{ij}=-\eta \frac{\partial E}{\partial w_{ij}}, \end{array}$$

(11) $$\begin{array}{c} \Delta \theta_{i}=-\eta \frac{\partial E}{\partial \theta_{i}}, \end{array}$$

where *η* represents the learning rate. The following equations are obtained.

(12) $$\begin{array}{c} \Delta w_{ki}=-\eta \sum_{P=1}^{P}\sum_{\mathrm{k=1}}^{l}\left(T_{k}^{P}-y_{k}^{P}\right)\cdot \psi \left(\delta_{k}\right)\cdot \beta_{i}, \end{array}$$

(13) $$\begin{array}{c} \Delta a_{k}=\eta \sum_{\mathrm{P=1}}^{P}\sum_{\mathrm{k=1}}^{l}\left(T_{k}^{P}-y_{k}^{P}\right)\cdot \psi \left(\delta_{k}\right), \end{array}$$

(14) $$\begin{array}{c} \Delta w_{ij}=\eta \sum_{\mathrm{P=1}}^{P}\sum_{\mathrm{k=1}}^{l}\left(T_{k}^{P}-y_{k}^{P}\right)\cdot \psi \left(\delta_{k}\right)\cdot w_{ki}\cdot \phi \left(\alpha_{i}\right)\cdot x_{j}, \end{array}$$

(15) $$\begin{array}{c} \Delta \theta_{i}=\eta \sum_{\mathrm{P=1}}^{P}\sum_{\mathrm{k=1}}^{l}\left(T_{k}^{P}-y_{k}^{P}\right)\cdot \psi \left(\delta_{k}\right)\cdot w_{ki}\cdot \phi \left(\alpha_{i}\right). \end{array}$$

IGA [19] is adopted and BPNN is optimized. The improved algorithm—IGA-BPNN prediction algorithm—is proposed. IGA is an optimization algorithm that combines Immune Algorithm immune theory (IA) and Simple Genetic Algorithm basic genetic algorithm (SGA) to complement each other. The main method is to use IGA to calculate the optimal weight and threshold of BPNN instead of updating it through BPNN itself. The IGA-BPNN algorithm flow is shown in Figure 4.

#### 2.2.2. BPNN Attribute Characteristics

The constructed mortality prediction model using BPNN is mainly using extracting the relevant feature indicators of patient information in the original data, scoring, and analysing to predict the mortality. Therefore, before the model performs prediction work, a feature set needs to be established. Fourteen materialized views have been created in the Oracle database. The names and meanings of the views are shown in Figure 5.

According to the materialized view in Figures 6 and 7, basic scoring features, critical scoring features, and 36 diagnosis and treatment attribute features are extracted. The basic and critical scoring characteristics are shown in Figure 6.

### 2.3. Design of Nursing Information Management System

#### 2.3.1. Patient Information Management Module

This module is mainly responsible for the management of basic personal information, medical information, and nursing information of patients in the ICU. The module provides four functions of adding, deleting, modifying, querying, and transferring patient information. The query function mainly realizes automatic acquisition of patient information by connecting to the HIS system. The architecture of the patient information management module is shown in Figure 7.

#### 2.3.2. Message Notification Module

The message notification module is mainly to provide news push for medical staff in neurosurgery ICU. When a new work schedule appears in the ICU, the administrator only needs to log in to the system, write the schedule notification in the corresponding text box, and select the relevant individual or group to push, to realize the differentiated push of messages. Push notifications are not limited to text, but can also be combined with pictures, sounds, and videos to make them more intuitive. The administrator can also set the urgency of the notification, and the system will present different display effects according to different settings. In order to prevent accidents caused by medical staff forgetting their tasks, the module provides the function of regular and repeated push. This function can be set to repeatedly push important notifications.

#### 2.3.3. Mortality Prediction Module

This module mainly uses the constructed BPNN model to predict mortality using the medical information data of critically ill patients in neurosurgery. After the doctor finds the patient's care information in the system, he sends a prediction request to the system. The BPNN model in the system is used to automatically extract the relevant feature indicators in the patient information data, and the mortality rate is predicted. After the prediction is over, the results are fed back to the client to assist the doctor in the analysis and diagnosis of the patient's condition. This will undoubtedly greatly improve the efficiency of the ICU and the success rate of treatment. The workflow of the mortality prediction module is shown in Figure 8.

#### 2.3.4. Account Information Management Module

This module mainly manages and maintains the account information of all users in the system. When medical staff register, the account default is the work number. The password, personal information, bound e-mail address, and contact information are set. This information can be deleted and changed in the system. If the password is forgotten, it will be retrieved or reset via e-mail or mobile verification. The system administrator can query, delete, modify, and freeze all accounts. The structure of the account information management module is shown in Figure 9.

#### 2.3.5. Authority Management Module

This module is mainly to provide the administrator with the function of assigning access and operation authority to others. All departments in the hospital, including neurosurgery, have different ranks and positions, and the corresponding scope of work and responsibilities are also different. Therefore, the administrator needs to manage the authority according to the actual situation of each department of the hospital. Different roles have different access and operation permissions in the system.

### 2.4. Mortality Prediction Model Test Method

#### 2.4.1. Selection of Data Set

Medical Information Mart for Intensive Care (MIMIC)-III data set [20] is selected to test the model. The MIMIC-III data set is a public data set established by the Computational Physiology Laboratory of Massachusetts Institute of Technology. It contains all the physiological monitoring data of more than 50,000 critically ill patients from 2001 to 2012. Among them, the data includes records and codes of the patient's vital signs, drug records, hospitalization information, experimental tests, and observation results and is stored in CSV format. In MIMIC-III, the relevant data in CSV format is downloaded. The data is deployed to the Oracle database management system and is named MIMIC.

#### 2.4.2. BPNN Structure

According to the established scoring feature set, the number of input layer nodes of BPNN is determined to be 17. The output data is the number of deaths and mortality of critically ill patients. Therefore, the number of nodes in the output layer of BPNN is 2. Using the determined number of nodes in the input layer and output layer of the model, the calculation equation for the number of nodes in the hidden layer shows that the range is within[5, 14]. The number of nodes in the hidden layer has a great influence on the training speed and accuracy of the model. Too many nodes will cause the network to converge slowly, and too few nodes will not guarantee the prediction accuracy of the model. Therefore, the model's predictions of Mean Square Error (MSE), Mean Absolute Error (MAE), and Root Mean Square Error (RMSE) under different hidden layer nodes are tested. The calculation of RMSE, MAE, and MSE is as follows:

(16) $$\begin{array}{c} RMSE=\sqrt{\frac{1}{n}\sum_{\mathrm{i=1}}^{n}{\left({\hat{y}}_{i}-y_{i}\right)}^{2}}. \end{array}$$

Among them, ${\hat{y}}_{i}$ is the predicted value; *y*_*i*_ is the actual value; and *n* is the total number of samples.

(17) $$\begin{array}{c} MAE=\frac{1}{n}\sum_{\mathrm{i=1}}^{n}\left|{\hat{y}}_{i}-y_{i}\right|\\ MSE=\frac{1}{n}\sum_{\mathrm{i=1}}^{n}{\left({\hat{y}}_{i}-y_{i}\right)}^{2}. \end{array}$$

The training parameter settings of the IGA-BPNN model are shown in Table 2.

#### 2.4.3. Specific Experimental Methods

Firstly, using the relevant indicators in the feature set, sample features are extracted from the MIMIC-III data set. Through sorting and summarizing, the sample set is constructed. The data from 2001 to 2010 is selected as the model training set, and the data from 2011 to 2012 is used as the test set for model performance testing. Secondly, the training set is used to train the model. Input the test set into the trained IGA-BPNN model to be predicted experiment. Finally, the Precision (*P*), Recall (*R*), and *F*1-score are used as evaluation indicators. At present, the more popular *K*-Nearest Neighbor (KNN) [21], Multilayer Perceptron (MLP) [22], and Random Forest (RF) [23] are selected for comparison and analysis with the model. The calculation equations of the three evaluation indicators are as follows:

(18) $$\begin{array}{c} P=\frac{TP}{TP+FP}, \end{array}$$

(19) $$\begin{array}{c} R=\frac{TP}{FN+TP}, \end{array}$$

where True Positive (*TP*) indicates that the prediction is positive, and the actual is also positive; False Positive (*FP*) indicates that the prediction is positive, but the actual is negative; True Negative (*TN*) indicates that the prediction is negative, and the actual is also negative; and False Negative (*FN*) indicates that the prediction is negative, and the actual is positive.

(20) $$\begin{array}{c} F1=\frac{2P\cdot R}{P+R}. \end{array}$$

### 2.5. System Performance Test Method

The database server, application server, and client server configuration in the system test are shown in Table 3.

The number of CPU cores in the system is 10, the number of service threads is 20, and there are 1000 requests per connection. When the system server is tested, the Net Assist network assistant is used to simulate the sending of data from multiple smart devices to simulate the real environment in which the system operates. Deploy 1 server, 8 simulated wireless infusion pumps and ECG monitors, and each simulated assistant runs 1024 concurrently. Meanwhile, the server is subjected to read and write operations, data transmission, and the number of requests per second and response time of the server under different numbers of concurrent threads.

## 3. Results and Evaluations

### 3.1. Effectiveness of the Proposed System Function Modules

#### 3.1.1. Login Page

The effect of the system login page is shown in Figure 10.

#### 3.1.2. Patient Information Management Module

The effect of the patient information management page is shown in Figure 11.

#### 3.1.3. Account Information Management Module

The effect of the account information management page is shown in Figure 12.

#### 3.1.4. Authority Management Module

The effect of the rights management page is shown in Figure 13.

### 3.2. Test Results of Mortality Prediction Model Using IGA-BPNN

#### 3.2.1. Determination of the Number of Hidden Layer Nodes

The prediction results of the model under different hidden layer nodes are shown in Figure 14.

Figure 14 shows that when the number of hidden layer nodes is 8, the model prediction error reaches the lowest and the performance reaches the best. Therefore, it is finally determined that the network structure of BPNN is 17 ∗ 8 ∗ 2.

#### 3.2.2. Comparison of Predictive Performance Test Results

The results of using different models to predict patient mortality are shown in Figure 15.

From the overall trend, the Precision, Recall, and *F*1 values of the constructed IGA-BPNN prediction model are all the highest. The predicted precisions of KNN, MLP, RF, and IGA-BPNN are 0.83, 0.65, 0.81, and 0.89, respectively, and the precision of the model is higher than other models by more than 7.2%. The Recall of the four models is 0.83, 0.65, 0.64, and 0.89, respectively, which is more than 7.2% higher than that of the model. The *F*1 values of the four models are 0.82, 0.66, 0.69, and 0.88, which are 7.3% higher.

In summary, the model has better predictive performance. BPNN also has the advantages of self-learning and self-organization, realizes the automation and intelligence of the prediction process, and is more suitable for the mortality prediction of critically ill patients in neurosurgery.

### 3.3. System Performance Test Results

The test results of the number of requests per second and the average response time of the system with different numbers of concurrent threads are shown in Figure 16.

In Figure 16, as the number of concurrent threads in the system increases, the number of requests processed per second by the system also increases exponentially. When the number of concurrent threads is less than 1024, the average response time of the system has been maintained at about 40 ms. After the number of concurrent threads is greater than 1024, although the average response time of the system also increases significantly, the impact of millisecond-level changes on the real-time response of the system is less obvious. Therefore, the system meets the requirements of high concurrency environment and has high performance.

## 4. Conclusion

The traditional nursing information management system can only manage the relevant information of patients but cannot analyze the data. In addition, the way of manually judging the patient's condition has problems such as strong subjectivity and low accuracy, which is not conducive to timely treatment of patients. Firstly, a mortality prediction model using IGA-BPNN is proposed. Secondly, a nursing information management system for critically ill patients in neurosurgery is designed. The IGA-BPNN prediction model is used as a part of the system to predict the mortality of critically ill patients. Finally, the experiment is designed to test the prediction model and the performance of the system. The results show that the Precision, Recall, and *F*1-score of the IGA-BPNN model for mortality prediction are 7.2%, 7.2%, and 7.3% higher than other prediction models, respectively. The comprehensive performance of the system during operation can reach the standard. The disadvantage is that only one data set is selected to verify the model, and the data type is relatively single and not representative. In the future, the scope of data selection needs to be expanded to further improve the model. The purpose of this research is to provide important technical support for the nursing information management of critically ill patients in neurosurgery and the intelligent analysis of the patient's condition.

In the future, the proposed system can be extended to automate various activities related to the doctors, such as the visits schedules. Additionally, what was advised to a particular patient during a visit should be described and incorporated in the extended version of the proposed model.

## Figures and Tables

**Figure 1:** Network architecture of the system.

**Figure 2:** BPNN structure diagram.

**Figure 3:** BP algorithm flow chart.

**Figure 4:** IGA-BPNN algorithm flow chart.

**Figure 5:** Materialized view.

**Figure 6:** Scoring feature set.

**Figure 7:** The architecture diagram of the patient information management module.

**Figure 8:** Workflow chart of the mortality prediction module.

**Figure 9:** Architecture diagram of account information management module.

**Figure 10:** The effect diagram of the system login interface.

**Figure 11:** The effect diagram of the patient information management interface.

**Figure 12:** The effect diagram of the account information management interface.

**Figure 13:** The effect diagram of the authorization management interface.

**Figure 14:** Model performance test results under different hidden layer nodes.

**Figure 15:** Comparison of mortality test results of different models.

**Figure 16:** Test results of system performance.

**Table 1:** Comparison of advantages and disadvantages of B/S and C/S.

	B/S structure	C/S structure
Advantage	Strong distribution, zero maintenance on the client side; simultaneous access by multiple users; easy to maintain, upgrade, and add new features; simple development and strong sharing; simple aspect of business expansion	Quick response; the operation interface is beautiful and diverse, which can meet the personalized requirements of users; higher security, suitable for high-security systems; strong business processing ability
Disadvantages	Low personalization; the program code is not separated logically, which is not conducive to reuse; slow response and poor coupling; system porting is difficult; security is low	Low resource utilization; clients need to be configured one by one, which is more complicated; client development and maintenance costs are high, and upgrades are difficult; the user group is fixed, and the scope of application is narrow; poor compatibility, high system configuration requirements

**Table 2:** Training parameter values of IGA-BPNN model.

Parameter	Numerical value
Training times	10000
Learning rate	0.5
Activation function	ReLU
Number of populations	2
Number of iterations	2
Crossover probability	0.7
Mutation probability	0.05

**Table 3:** Environment required for system testing.

Project	Configure
Operating system	Windows 10
Central processing unit (CPU)	Intel Core i7-7700 3.60 GHz
Random access memory (RAM)	8 GB
Hard disk	500 GB

## Data Availability

The data that support the findings of this study are available from the corresponding author upon reasonable request.

## References

[1] Ni L., Xue P., An C. (2021 Nov 28). Establishment of normal range for thromboelastography in healthy middle-aged and elderly people of weihai in China. *Journal of Healthcare Engineering*.

[2] Zheng L., Feng H., Yin L. (2021 Oct 27). Study on the correlation factors of tumour prognosis after intravascular interventional therapy. *Journal of Healthcare Engineering*.

[3] Yeh A., Pietras C., Wallenstein D., Hu P. (2019). End of life in the neurological intensive care unit: is extubating to comfort care comfortable?. *Journal of Pain and Symptom Management*.

[4] Jebraeily M., Rahimi B., Fazlollahi Z. Z., Afshar H. L. (2019). Using SERVQUAL model to assess hospital information system service quality. *Hormozgan Medical Journal*.

[5] Cao Y., Zhu H. (2020). Research on digital information system construction and intelligent management of clinical pediatric nursing in hospital. *Journal of Medical Imaging and Health Informatics*.

[6] Shahmoradi L., Ebrahimi M., Shahmoradi S., Farzanehnejad A., Koolaee M. H. (2020). Usage of standards to integration of hospital information systems. *Frontiers in Health Informatics*.

[7] Shojaei Baghini M., Baniasadi N. (2020). Evaluation of nursing information system: nurses’ perspectives. *Applied Health Information Technology*.

[8] Sallow A. B., Dino H. I., Ageed Z. S., Mahamood M. R., Abdulrazzaq M. B. (2020). Client/Server remote control administration system: design and implementation. *Int. J. Multidiscip. Res. Publ*.

[9] Gong Y. (2018). Design and implementation of English for academic purpose online learning system based on browser/server framework. *International Journal of Emerging Technologies in Learning (iJET)*.

[10] Wang T., Li N., Li H. (2021). Design and development of human resource management computer system for enterprise employees. *Plos one*.

[11] Li A. (2020). Impact of data statistics on the execution plan of the oracle database. *Journal of Physics: Conference Series*.

[12] Li T., Sun J., Wang L. (2018). An intelligent optimization method of motion management system using BP neural network. *Neural Computing & Applications*.

[13] Wang J., Shi P., Jiang P., Hu J., Qu S. (2017). application of BP neural network algorithm in traditional hydrological model for flood forecasting. *Water*.

[14] Wu B., Han S. J., Xiao J., Hu X., Fan J. (2016). Error compensation using BP neural network for airborne laser ranging. *Optik - International Journal for Light and Electron Optics*.

[15] Lin Y. C., Chen D. D., Chen M. S., Chen X.-M., Li J. (2018). A precise BP neural network-usingline model predictive control strategy for die forging hydraulic press machine. *Neural Computing & Applications*.

[16] Cheng S., Wu Y., Li Y., Yao F., Min F. (2021). TWD-SFNN: three-way decisions with a single hidden layer feedforward neural network. *Information Sciences*.

[17] Lin S. (2021). Financial performance management system and wireless sharing network optimization of listed enterprises under BPNN. *Mobile Information Systems*.

[18] Lv Y., Liu W., Wang Z., Zhang Z. (2020). WSN localization technology using hybrid GA-PSO-BP algorithm for indoor three-dimensional space. *Wireless Personal Communications*.

[19] Katoch S., Chauhan S. S., Kumar V. (2021). A review on genetic algorithm: past, present, and future. *Multimedia Tools and Applications*.

[20] Dan-Ni W. N. A. G., Li-Dian H. U. A., Zhi-Guo P. A. N. (2021). The impact of body mass index on the prognosis in sepsis patients: a retrospective analysis on account of the large clinical database MIMIC-III. *Medical Journal of Chinese People’s Liberation Army*.

[21] Abu Alfeilat H. A., Hassanat A. B., Lasassmeh O. (2019). Effects of distance measure choice on k-nearest neighbor classifier performance: a review. *Big Data*.

[22] Heidari A. A., Faris H., Aljarah I., Mirjalili S. (2019). An efficient hybrid multilayer perceptron neural network with grasshopper optimization. *Soft Computing*.

[23] Zamani M. (2019). PM2. 5 prediction using random forest, XGBoost, and deep learning using multisource remote sensing data. *Atmosphere*.

